# A Clinical Analysis and Literature Review of Six Cases with Primary Pulmonary Lymphoepithelioma-Like Carcinoma

**DOI:** 10.1155/2022/1086697

**Published:** 2022-04-29

**Authors:** Lingyan Ye, Dinghai Luo, Haiyan Li, Haihong Zheng, Susu He, Ling Lin, Yicheng Fang, Junhui Ye, Chengshui Chen

**Affiliations:** ^1^Department of Respiratory Medicine, Taizhou Hospital of Zhejiang Province affiliated to Wenzhou Medical University, Linhai, Zhejiang, China; ^2^Department of Gastroenterology, Taizhou Hospital of Zhejiang Province Affiliated to Wenzhou Medical University, Linhai, Taizhou, China; ^3^Department of Pathology, Taizhou Hospital of Zhejiang Province affiliated to Wenzhou Medical University, Linhai, Zhejiang, China; ^4^Department of Radiology, Taizhou Hospital of Zhejiang Province affiliated to Wenzhou Medical University, Linhai, Zhejiang, China; ^5^Department of Respiratory Medicine, The People's Hospital of Sanmen, Taizhou, Zhejiang, China; ^6^Department of Respiratory and Critical Care Medicine, The First Affiliated Hospital of Wenzhou Medical University, Wenzhou, Zhejiang, China

## Abstract

**Methods:**

The clinical data of six patients with primary pulmonary lymphoepithelioma-like carcinoma treated in Zhejiang Taizhou Hospital of Taizhou Enze Medical Center (Group) from May 2014 to December 2018 were summarized and analyzed. Combined with the relevant literature, the primary pulmonary lymphoepithelioma-like carcinoma was analyzed retrospectively.

**Results:**

The main manifestations of six patients were respiratory symptoms, and cough was the most common. The imaging features of six patients were mainly round-like high-density mass shadow or nodule shadow. All patients were diagnosed by pathology. Microscopically, the cancer cells were nested, with large nuclei and vacuoles and abundant lymphocyte infiltration in the tumor stroma. The positive rates of EBER, p63, CK5/6, and Ki-67 were high, and TTF-1 was negative. Five patients received surgical treatment. One patient developed brain metastasis 12 months after operation and received craniocerebral radiotherapy. The other patients did not receive radiotherapy and chemotherapy, and one patient did not receive treatment. After follow-up, four patients survived so far, the longest survival time was 82 months, one patient lost follow-up, and one patient died of lung metastasis 24 months after operation.

**Conclusion:**

Primary pulmonary lymphoepitheliomatoid-like carcinoma is a rare lung malignant tumor, whose pathogenesis is related to Epstein-Barr virus infection. The clinical manifestations are nonspecific, but with unique pathological characteristics. Surgical resection is the proper treatment for early-stage patients, and comprehensive treatment with surgery as the main treatment is suitable for late-stage patients. The prognosis is good.

## 1. Introduction

Lymphoepithelioma-like carcinoma can occur in organs of foregut origin such as stomach, parotid gland, thymus, and lung, among which pulmonary lymphoepithelioma-like carcinoma is the most rare [1]. Primary pulmonary lymphoepithelioma-like carcinoma (PPLELC) is a rare malignant tumor in the lung, belonging to a subtype of large cell lung cancer; the incidence rate is only 0.92% [2] of lung cancer. Previous studies have suggested that Epstein-Barr virus (EBV) infection may be closely related to its onset [3]. The disease is common in Asian populations, and the incidence is mainly young and nonsmoking patients [4]. So far, only more than 200 cases of primary pulmonary lymphoepithelioma-like carcinoma have been reported, and the clinical manifestations are nonspecific; most of them are cough, expectoration, hemoptysis, chest tightness, chest pain, or low fever [5]. There is no significant difference with the clinical manifestations of other lung diseases, which is very easy to be misdiagnosed or missed. Many cases have been reported to be misdiagnosed as lung squamous cell carcinoma [6, 7]. At present, there is no definite treatment guideline for primary pulmonary lymphoepithelioma-like carcinoma; most of them follow the treatment scheme of non-small-cell lung cancer. Fan et al. [8] reported the feasibility of immunotherapy. Because it is relatively rare, the literature on primary pulmonary lymphoepithelioma-like carcinoma is mostly reported by individual cases and rarely involves the overall understanding of it. This paper collected the clinical data, clinical manifestations, imaging features, pathological features, treatment methods, and prognosis of six patients with primary pulmonary lymphoepithelioma-like carcinoma in our hospital, combined with the relevant literature, so as to provide direction for the in-depth study of this rare type of lung cancer and explore more effective treatment methods.

## 2. Methods

### 2.1. Participants

Six patients with PPLELC treated in Taizhou Hospital of Zhejiang Enze medical center (Group) from May 2014 to December 2018 were selected. The data of gender, age, smoking history, past medical history, clinical symptoms, imaging findings, tumor location, tumor size, staging, treatment method, and prognosis were collected and analyzed through electronic medical records.

### 2.2. Diagnosis

All patients were confirmed by pathology. One case underwent lung biopsy under CT positioning, and five cases underwent surgical thoracoscopic resection. All tissue samples were routinely detected by HE staining combined with immunohistochemical staining and EBV small RNA (EBER) by in situ hybridization, which met the diagnostic criteria of primary lung LELC [4], except for lung metastasis of nasopharyngeal carcinoma. Immunohistochemical staining: six specimens were fixed with 3.7% neutral formaldehyde solution, routine paraffin dehydration, embedding, sectioning, HE staining, and light microscopic observation. The antibodies used were broad-spectrum cytokeratin (ckpan), P40, p63, CD3, CD8, and CD20 purchased from Fuzhou Maixin Biotechnology Development Co., Ltd. Immunohistochemical steps: sheep antimouse/antirabbit Power Vision two-step method, incubate at room temperature for 20 minutes, rinse with PBS buffer for 3 minutes, three times in total, add an appropriate amount of DAB chromogenic solution, rinse at room temperature for 5 minutes, rinse with running water, contrast staining with hematoxylin for 1 minutes, and then dehydrate with gradient ethanol, transparent, seal, and read the film. EBER in situ hybridization: 21 samples were fixed with 3.7% neutral formaldehyde solution, conventional paraffin dehydration, embedding, slicing, baking, dewaxing, digestion, dehydration and drying, probe addition, sealing, hybridization (hybridization with Abbott's automatic hybridization instrument), primary antibody incubation, secondary antibody incubation, mixture incubation, color development, comparative staining, dehydration, transparency, sealing, and then read the film. The TNM staging of patients is based on the eighth edition of international lung cancer staging formulated by the lung cancer research association [9].

### 2.3. Treatment Plan

Five cases were treated surgically, all of them underwent thoracoscopic radical resection of lung cancer, of which one case had brain metastasis 12 months after operation and received radiotherapy, and the other four patients did not receive postoperative radiotherapy and chemotherapy; one case was not treated. All five patients were followed up by lung CT.

### 2.4. Follow-Up

Six patients were followed up by outpatient or telephone. The follow-up time was up to February 28, 2021, and one patient lost the follow-up. Survival (OS) is defined as the time from diagnosis to death or the deadline of follow-up. For patients who lost follow-up, the survival time ended to the last follow-up.

### 2.5. Results

The clinical data of six patients with PPLELC are shown in Table 1. Among the six patients, there were four males and two females, aged 55-74 years, with a median age of 64.6 years. One patient had a history of smoking, three patients had a history of hypertension, and one patient had a history of diabetes. There were four cases with cough and expectoration symptoms, including one case with blood in sputum, one case with fever, and two cases without any symptoms or found in physical examination. The lung CT findings of six patients were round-like high-density mass or nodule (Figures 1–3), with clear boundary; some of them were shallow lobulated, with a diameter of 1.0-6.4 cm. There were five cases of unilateral lesions, one case of bilateral lesions, four cases of lesions located in the right lung, and two cases in the left lung. No air bronchial sign, cavity, calcification, and other signs were found in the masses of all patients. All the six patients were pathologically confirmed as PPLELC. Histologically, it can be seen that in the background of diffuse distribution of mature lymphocytes, undifferentiated or poorly differentiated cancer cells were arranged in strip, nest, or single scattered distribution. The cancer cells were oval or polygonal in shape, with large nuclei and vacuoles and obvious nucleoli (Figure 4). The mitotic images were different. Immunohistochemical staining showed that cytokeratin (CK) was positive, TTF-1 was negative, p63 was positive in five cases, and the expression rate of Ki-67 was 40-70%. EBER in situ hybridization was positive in four cases (66.7%) (Figure 5). Among the six patients, three cases were in stage I, two cases were in stage III, and one case was in stage IV. After follow-up, four of the six patients have survived so far, including one case with brain metastasis 12 months after operation, and still survived after craniocerebral radiotherapy. The survival time of the four patients was more than 3 years, and the longest OS was 82 months; one case was lost to follow-up after 3 months, and one case died of intrapulmonary metastasis after 24 months.

## 3. Discussion

Primary pulmonary lymphoepithelioma-like carcinoma (PPLELC) is a rare malignant tumor of the lung. Bégin et al. [1] first reported LELC of the lung in 1987. In the edition of 2015 WHO histological classification of lung cancer, LELC was classified into other unclassified cancer groups in non-small-cell lung cancer [10]. PPLELC mostly occurs in nonsmokers [4]. In this study, smoking patients account for 16.7%, which indicates that smoking may not be significantly related to its pathogenesis. Many studies believe that the pathogenesis of LELC is closely related to EB virus infection [11, 12], but the specific mechanism is not clear. According to relevant clinical reports [13], about 75% of patients with PPLELC tested positive for EB virus. In this study, four cases (66.7%) were EBER positive by in situ hybridization, which was consistent with the reports of Javed [13] and also explained the correlation between EB virus infection and PPLELC. Unfortunately, we did not carry out EB virus serological examination in the six patients.

PPLELC patients lack specific clinical manifestations, mainly manifested as respiratory symptoms such as cough, expectoration, and chest pain. Ho et al.'s [4] research showed that 47% of patients presented with cough at the first diagnosis. Mo et al.'s [14] research found that about 20%-35% of patients had no symptoms at the beginning of onset. In this study, two patients(33.3%) were asymptomatic. Four patients showed cough, expectoration, and blood in sputum, which were similar to the clinical symptoms of other lung diseases, so it was difficult to diagnose by clinical symptoms. Ooi et al. [15] considered that PPLELC had unique imaging characteristics, most of the early lesions were close to the pleura, and the late lesions were easy to invade the bronchus and large vessels. Many studies have shown that [16–18] the chest imaging characteristics of PPLELC were mainly peripheral single mass or nodule, mostly single focus. Most of the lesions occur in the lower lobe of the lung and close to the mediastinal pleura. Most of the masses or nodules were smooth, round, or irregular at the edge, without obvious hair prick sign, cavity, and calcification. Enhanced scanning showed that the lesions were more evenly enhanced, and a few parts can be seen without enhanced liquefaction necrosis. In this study, the lung CT findings of six patients mainly showed round-like high-density mass or nodule shadow, with clear boundary and no obvious burr. Except for one case with intrapulmonary and pleural metastasis, the rest were single lesions. The imaging findings were consistent with the above study.

At present, the diagnosis of PPLELC still depends on the results of histopathology and immunohistochemical staining. The pathological diagnosis of PPLELC needs to be confirmed by fiberoptic bronchoscopy biopsy, percutaneous lung biopsy, and surgical pathology. Histologically, the typical PPLELC is similar to the dumb type of vesicular nuclear cell carcinoma of undifferentiated nasopharyngeal carcinoma. Under the microscope, the tumor cells are arranged in nests or irregular clusters. The cancer nucleus are round, oval, or slender, with obvious atypia, clear nucleoli, vesicular nucleus, and medium amount of cytoplasm [19]. A large number of plasma cells or mature lymphocytes are seen in the stroma, and fibrous tissue proliferation is obvious [20]. The pathology of six patients in this study was consistent with the typical LELC manifestations in the literature. In terms of immunohistochemistry, PPLELC did not express glandular epithelial markers (TTF-1, CK20, and Napsin A) but highly expressed squamous epithelial markers (CK5/6, p63, and P40) [21]. In this study, CK was positive in all six patients, TTF-1 was negative, and p63 and Ki-67 were positive in five patients, indicating that PPLELC may have characteristics similar to squamous epithelial differentiation.

As PPLELC is rare in clinic, there is no unified treatment scheme at present. Lin et al. [22] suggested that early surgical resection of PPLELC is feasible. Liang et al. [23] suggested that no lymph node metastasis and complete tumor resection can enable patients to obtain better survival rate. For patients with locally advanced PPLELC, concurrent radiotherapy and chemotherapy are the main treatments, while patients with stage IV mostly choose comprehensive treatment based on surgery [24–26]. At present, platinum-based dual drug-combined chemotherapy is the first-line treatment for PPLELC. In this study, five patients were treated according to the principle of non-small-cell lung cancer treatment, three patients were stage I and underwent thoracoscopic radical resection of lung cancer, two patients were stage IIIa and underwent thoracoscopic radical resection of lung cancer combined with lymph node dissection; one of the five patients had brain metastasis one year after operation and received radiotherapy, but the other four patients and one patient in phase IV did not receive radiotherapy and chemotherapy, so the efficacy of radiotherapy and chemotherapy could not be evaluated. Chan A. et al. [24] observed the sensitivity of 7 patients with PPLELC to chemotherapy and found that 5 patients (71.4%) were sensitive to chemotherapy. Lin et al. [26] found that radiotherapy also had a certain sensitivity. Previous reports [22, 23, 27] have shown that PPLELC had a better prognosis than other non-small-cell lung cancer, and tumor recurrence and necrosis are poor prognostic factors for survival. According to Liang et al. [23], the median survival time of patients with PPLELC was 31.55 months, and the 2-year and 5-year overall survival rates were 88% and 62%, respectively. The survival time of four patients in this study was more than 36 months, and the longest was 82 months. The follow-up data were basically consistent with the literature. Targeted therapy and immunotherapy are the research hotspots of lung cancer. A number of studies [21, 28–30] showed that the mutation rates of EGFR and ALK genes in patients with PPLELC were significantly lower than those in non-small-cell lung cancer patients, and the benefit of targeted therapy was small, but 63.3%-75.8% of patients with PPLELC expressed PD-L1. Fan et al. [8] showed that PPLELC had a higher expression rate of PD-L1 than conventional NSCLC, and the disease control rate of receiving PD-L1 inhibitor reached 90.9%. However, the clinical therapeutic effect of PPLELC on immunotherapy needs to be further studied in more cases. Unfortunately, none of our six patients were tested for driver gene and PD-L1, and we were unable to know the mutation gene and PD-L1 expression rate.

There are still some defects in our study. Firstly, we are a single center retrospective study. Some clinical data are incomplete, and the significance of the data may not be enough because of the small number of cases. At the same time, all patients were not tested for driver gene and PD-L1, nor were they treated with PD-L1, so they were unable to know the effectiveness of immunotherapy.

In summary, primary pulmonary lymphoepithelioma-like carcinoma is rare in clinic. Its incidence is closely related to EB virus. There is no specificity in clinical symptoms and imaging manifestations. The diagnosis needs to be based on pathological results. At present, there is no standardized treatment scheme. Surgical resection is the main treatment for early patients, and immunotherapy may be beneficial to advanced or late patients. At present, more prospective studies are still needed to understand the best treatment scheme and long-term survival of the disease.

## Figures and Tables

**Figure 1:** The soft tissue mass in the right upper lobe of the lung has clear boundary, uneven density, and vascular invasion, with intrapulmonary and pleural metastasis.

**Figure 2:** The nodule in the right lower lobe of lung, with clear margin.

**Figure 3:** The nodule in the right middle lobe of the lung, with shallow lobulated.

**Figure 4:** In diffuse lymphocytes, the cancer cells are arranged in nests and scattered, oval or polygonal, with large, vacuolar nuclei and prominent nucleoli (high magnification with HE staining).

**Figure 5:** Eber in situ hybridization positive (in situ hybridization low magnification).

**Table 1:** The clinical data of 6 patients with PPLELC.

Patient	Sex	Age	Smoking history	Clinical symptoms	Tumor			EBER	Treatment	OS (month)
					Position	Size	Stage			
1	Male	64	None	None	Right lower lobe of lung	1.7∗1.8 cm	T1bN0M0 IA	+	Surgery	67
2	Female	59	None	Cough and expectoration	Right middle lobe of lung	1.0∗1.4 cm	T1bN0M0 IA	+	Surgery	41
3	Female	74	None	Cough and fever	Right upper lobe of lung	6.4∗4.8 cm	T4N2M1a IVA	+	None	3
4	Male	66	Yes	Cough and blood in sputum	Left upper lobe of lung	3.3∗2.5 cm	T2aN2M0 IIIA	—	Surgery+brain radiotherapy	60
5	Male	70	Yes	Cough and expectoration	Right middle lobe of lung	5.2∗4.4 cm	T3N1M0 IIIA	—	Surgery	24
6	Male	55	None	None	Left lower lobe of lung	3.4∗2.5 cm	T2aN0M0 IB	+	Surgery	82

## Data Availability

Study data are available from the corresponding author.
